RETRACTED

# Correlation between Breast Ultrasound Microcalcification and the Prognosis of Breast Cancer

**DOI:** 10.1155/2021/6835963

**Published:** 2021-11-29

**Authors:** Shanshan Xue, Qiaoling Zhao, Minghui Tai, Ning Li, Yun Liu

**Affiliations:** ^1^Department of Ultrasound Medicine, The First Affiliated Hospital of Xi'an Jiaotong University, Xi'an, Shaanxi Province 710061, China; ^2^Department of Ultrasound, Wuhan Red Cross Hospital, Wuhan, Hubei Province 430015, China

## Abstract

Breast cancer is a common gynecological disease, and its incidence and mortality are higher than those of other common malignant tumors. Breast ultrasound technology is a new surgical method, which has the advantages of reducing postoperative complications, improving the quality of life of patients, and improving the prognosis of patients. Breast microcalcification is a new method for the treatment of tumors. Its mechanism is that the proliferation of breast cancer cell walls increases the inflammatory factors in the cancer tissues and enhances the formation of tumors and peripheral vascular thrombosis. Breast microcalcification in the treatment of breast cancer patients will have a more significant impact compared to ordinary antibiotics alone. For this reason, the microcalcification performance of breast ultrasound is worthy of study, and related research on prognosis is also indispensable. The purpose of this study is to improve the understanding of the ultrasound manifestations of breast cancer microcalcification and the prognosis of breast cancer. This article mainly applied statistical analysis as well as experimental and survey methods to conduct breast ultrasound examination on 100 patients and analyzed the ultrasound manifestations of breast cancer MCs from three aspects: location, shape, and distribution. The experimental results show that there is no correlation between the location and distribution of breast cancer MCs and the diameter of the cancer foci, but there is a certain correlation between the morphology (non-gravel-like calcification) and the diameter of the cancer foci (>5 cm). Among them, HER-2 overexpression accounted for 11.9% in the grit-like MCs group and 51% in the non-grit-like MCs group.

## 1. Introduction

Breast tumor is a serious disease that endangers human health and life safety. Its incidence rate remains high and it has become a topic worthy of attention in the world. The histological origin of breast cancer is mostly derived from ductal and acinar epithelial cells of various grades of the breast, and a very small number are derived from breast mesenchymal cells. The lesion develops from normal epithelial hyperplasia to atypical hyperplasia. If no intervention is given, it can gradually progress to carcinoma in situ, early invasive carcinoma to invasive carcinoma. Pathological indicators such as tumor size, axillary lymph node metastasis, and histological grade are the most effective and feasible reference factors for evaluating the prognosis of breast cancer. After the microcalcification is released in the tumor, the cell wall proliferates obviously and shows a trend of gradual enhancement and weakening of hemolytic function. The early detection rate of breast cancer is increasing year by year. Breast ultrasound microcalcification has a significant effect in the treatment group. Compared with conventional chemotherapy, it can significantly improve the immune level of lymphocytes, bone marrow, endoplasm, and other tissues after surgery. Breast microcalcification can affect the prognosis of patients. Through research, it is found that there is no significant difference in ultrasound time between the treatment group and the chemotherapy group. As patients age and more weight is gained, the infection rate in the operating room increases, and the incidence of mastitis within 1 hour before surgery is on the rise. The symptoms of breast cancer can be varied, including breast lumps, breast pain, nipple discharge, erosion or skin depression, and axillary lymph node enlargement. The majority of breast cancer is invasive growth and the boundary is not clear. Some can be flat, the surface is not smooth, and there is a nodular feeling. However, it should be noted that the smaller the mass, the less obvious the previously mentioned symptoms. Moreover, a few special types of breast cancer may be inflated due to less invasive growth. They are smooth, active, and well defined and are not easy to distinguish from benign tumors.

RETRACTED

There are many conclusions about the correlation between the microcalcification manifestations of breast ultrasound and the prognosis of breast cancer. For example, Zhou Chengxiang retrospectively analyzed the breast imaging reports and data system ultrasound signs of breast cancer patients and explored the correlation between noninvasive ultrasound examination and the biological indicators of breast cancer molecular classification. It is concluded that the BI-RADS ultrasound signs of breast cancer have a certain diagnostic value in judging its molecular classification. Understanding the typical ultrasound signs of each molecular classification of breast cancer can help sonographers diagnose breast cancer earlier and more accurately [1]. Zhu Yangyang explored the correlation between the features of conventional ultrasound (US) and contrast-enhanced ultrasound (CEUS) of breast cancer and the expression level of HER-2. The results show that there are differences in the maximum diameter and microcalcification of US lesions among different expressions of HER-2. CEUS enhances uniformity, and there are differences in the different expressions of HER-2 in vascular nourishment and lesion enlargement after angiography. The peak intensity of TIC parameters is different from HER-2. The expression is related, the cut-off value is 9.045, the area under the curve is 0.704, the sensitivity is 91.2%, and the specificity is 64.2%; the previously mentioned statistically significant indicators are scored. US and CEUS are feasible methods to predict the expression of HER-2 gene in breast cancer and provide a basis for clinical treatment [2]. Li Dongqin explored the relationship between breast cancer microcalcification and the expression levels of estrogen receptor, progesterone receptor, and human epidermal growth factor receptor-2 (HER-2). The features of breast cancer mammography microcalcification can predict the expression of prognostic factors in breast cancer patients and provide certain help for the selection of breast cancer treatment options [3]. A variety of factors can lead to breast calcification, such as tissue degeneration, necrosis, and calcium salt deposition. Some tumors secrete substances containing calcium salt and calcify perivascular tissues. Analyzing the shape, number, and location of calcification and its relationship with surrounding structures is of great help to identify the nature of lesions. Simple breast calcification generally has no clinical discomfort, which is mainly the clinical manifestation of primary diseases, including breast swelling, pain, nipple overflow, or breast mass.

This article mainly discusses breast cancer, breast ultrasound technology, microcalcification manifestations, and prognostic factors in detail. First of all, this article starts with a simple introduction to breast cancer, studies the screening methods of breast cancer, analyzes the characteristics of breast cancer, and explains some current treatment methods for breast cancer. Secondly, it states the reasons for the use of ultrasound technology, the noise reduction method of ultrasound image formation, image segmentation, and feature extraction and explains its existing problems. Thirdly, this article studies microcalcification, firstly to understand the definition and secondly to analyze the relationship between microcalcification and mammary glands. Finally, the prognostic factors and indicators are analyzed and studied, and corresponding conclusions are drawn. The morphology of calcification is of great significance to distinguish between benign and malignant lesions. It is found that (1) coarse granular, eggshell, irregular mass, and orbital calcification mostly occur in benign lesions and (2) needle tip, small rod, bifurcation, cluster, and sediment calcification mostly occur in malignant lesions.

RETRACTED

## 2. Materials and Methods

### 2.1. Introduction to Breast Cancer

The appearance of any tumor is a change in molecular biological behavior through gene deletion and mutation, resulting in a mass-like tissue, producing abnormal physical changes that can be detected by imaging, and then forming individual appearance and internal subjective changes. The occurrence of breast cancer is the result of a combination of many factors [4, 5].

#### 2.1.1. Breast Cancer Screening Methods

Imaging examination has the characteristics of noninvasiveness, repeatability, and high precision. Medical imaging technology enables doctors to discover tumors in time, providing a reference for medical imaging and clinical diagnosis and diagnosis of breast tumors. Breast cancer is mainly dependent on mammography, MRI, CT, ultrasound, and so on. Ultrasonography is widely used in clinical practice because of its economic value, no radiation, and simple operation. With the development of ultrasound medical diagnosis and treatment technology, contrast-enhanced ultrasound came into being [6, 7].

#### 2.1.2. Features of Breast Cancer

1. Tumor morphology: lobulated or irregular mass, with irregular or ridged edges
2. Improved features: uneven enhancement within the lesion or ring-shaped enhancement at the edge
3. Dynamic gain scanning display, the early gain that reaches the peak within 3 minutes; the timing waveform is type III or type II

Compare the correlation of these imaging parameters with pathological and molecular biological indicators, determine the rules of their mutual influence, and study their application in assessing the prognosis of breast cancer [8, 9].

#### 2.1.3. Breast Cancer Treatment

At present, surgery is the mainstay, supplemented by comprehensive treatment concepts such as chemotherapy, radiotherapy, endocrine therapy, and targeted therapy. For different breast cancer patients, according to tumor lymph node metastasis, histological grade, pathological staging, molecular classification, etc., a variety of comprehensive treatment plans are adopted to reduce the recurrence rate, survival rate, and quality of life of patients [10].

Besides, targeted therapy is a treatment method for the identified carcinogenic site at the cellular and molecular level (the site can be a protein molecule in tumor cells or a gene fragment). Corresponding therapeutic drugs can be designed. When drugs enter the body, they will specifically select carcinogenic sites to combine and act, so as to make tumor cells die specifically without affecting normal tissue cells around the tumor. Therefore, molecular targeted therapy is also known as “biological missile.”

RETRACTED

### 2.2. Breast Ultrasound Technology

#### 2.2.1. Reasons for Using Ultrasound Technology

Breast tumor is a common disease among women in today's society. Early detection, early diagnosis, and early treatment are the principles of breast cancer prevention and treatment. Ultrasound imaging technology has the characteristics of wide adaptability, low price, no radiation, rapidness, and noninvasiveness. It can not only obtain soft tissue images without using contrast agents but also perform three-dimensional assessment of early tumor lesions and staging of malignant tumors. Preoperative evaluation and prognosis play an important role and are gradually becoming an important tool for early detection of breast tumors [11, 12].

#### 2.2.2. Ultrasonic Technology Image Processing

In the ultrasound image preprocessing part, the experiment comparatively analyzed the noise suppression effect of some commonly used filter models in ultrasound image processing and selected the filter to remove noise, while retaining the anisotropic diffusion model to eliminate speckle noise.

#### 2.2.3. Image Segmentation Method

In the segmentation of tumor boundary of breast ultrasound images, a semiautomatic segmentation algorithm based on graph cut theory and level set model based on distance regularization is first proposed. Next, an automatic breast ultrasound tumor segmentation algorithm based on Otsu threshold and improved CV model is proposed. The rough segmentation result is taken as the initial contour, and the improved CV model is used to develop it, and the final segmentation result is obtained.

The basic idea of the threshold image segmentation method based on wavelet transform is that, firstly, the histogram of the image is decomposed into different levels of wavelet coefficients by dyadic wavelet transform, and then the threshold is selected according to the given segmentation criteria and wavelet coefficients, and finally the image segmentation area is marked by the threshold. The local transform in spatial and frequency domain can effectively extract information from the signal and carry out multiscale analysis of the function or signal through the operation functions such as expansion and translation, which solves many problems that cannot be solved by Fourier transform. Because it is frequency domain operation, it is not sensitive to noise.

#### 2.2.4. Feature Extraction

In the part of breast tumor feature extraction, it combines the parameters commonly used in clinical diagnosis and the breast image report data system. In order to better identify the features with strong class distinction, this paper introduces the concept of class distance, selects the feature combination with the best classification ability according to the class distance between benign and malignant tumor features, and classifies subsequent tumors.

RETRACTED

Edges are pixels that make up the boundary (or edge) between two image regions. Generally, the shape of an edge can be arbitrary and may also include intersections. In practice, edges are generally defined as a subset of points with large gradients in the image. Some commonly used algorithms also connect the points with high gradient to form a more perfect description of the edge.

#### 2.2.5. There Is a Problem

Although ultrasound image recognition technology can effectively detect breast tumors, the structural differences between ultrasound imaging machines and human tissues pose major challenges to the segmentation and feature extraction of ultrasound images of breast tumors:

1. Affected by imaging equipment and mechanisms, there is a lot of speckle noise in ultrasound images, which makes the image signal-to-noise ratio and contrast low, and the edges become blurred.
2. There is a difference in acoustic impedance between human organs and tissue structures, and the ultrasound beam forms reflection, refraction, and scattering, which reduces the quality of ultrasound images and even produces artifacts.
3. There is tumor infiltration effect in breast ultrasound images; that is, tumors often invade surrounding normal tissues, making tumors very similar to surrounding normal tissues and difficult to distinguish.

The purpose of breast tumor ultrasound image segmentation is to extract the tumor contour boundary representing the lesion area in the image, so as to obtain the position and contour characteristics of the tumor. However, due to the inherent shortcomings of high speckle noise, low contrast, and blurred borders in breast ultrasound images, it brings about difficulties to the accurate segmentation of ultrasound images. Most of the existing segmentation algorithms for breast tumor ultrasound images are semiautomatic; that is, the region of interest is animated by hand and then automatically segmented by a computer. The semiautomatic segmentation method has made significant progress, reducing the workload of doctors. However, because breast tumors vary in size and shape, the boundaries are not clear, and even if the same patient is scanned by different ultrasound equipment, the results may not be the same. Therefore, a high-efficiency and high-accuracy automatic segmentation algorithm for breast tumor ultrasound images is a difficult point in breast ultrasound research.

RETRACTED

#### 2.2.6. Image Denoising

The Gaussian function has rotational symmetry and monotonic decline. The Gaussian filter has an obvious effect on removing the noise that obeys the normal distribution in the image. The Gaussian function has the same scale on the horizontal axis and the vertical axis and belongs to isotropic filtering. The function expression is shown in the following formula:

(1) $$\begin{array}{c} H\left[i,k\right]=d^{-\left(i^{2}k^{2}\right)/2\beta^{2}}. \end{array}$$

Mean filtering, median filtering, and Gaussian filtering are all isotropic diffusion models. The main idea of anisotropic diffusion filtering is to set different distribution coefficients in different directions. The diffusion equation is

(2) $$\begin{array}{c} \left\{\begin{array}{c} \frac{\ell I}{\ell p}=yis\left[x\left(a,b,p\right)\cdot \nabla I\right.\\ I\left(p=0\right)=I_{0} \end{array}\right\}. \end{array}$$

In addition, the mean filter itself has inherent defects; that is, it cannot protect the image details well. While denoising the image, it also destroys the details of the image, which makes the image blurred and cannot remove the noise points well. The median filtering method is very effective in eliminating salt and pepper noise and plays a special role in the phase analysis and processing of optical measurement fringe images.

#### 2.2.7. Image Segmentation

Ultrasound tumor image segmentation is a key component of the breast tumor ultrasound image CAD system. The quality of the segmentation effect directly affects the accuracy of subsequent feature extraction and the accuracy of classification.

The image segmentation algorithm based on graph theory maps the image to an undirected graph *H *=* *(*W*, *F*) and transforms the image segmentation problem into a graph optimization problem. Each pixel in the image corresponds to a vertex of the graph. In order to express the difference of each edge, a weight *w* is assigned to each edge, which is determined by the following formula:

(3) $$\begin{array}{c} {\text{w}}_{ik}=\left|I\left(s_{i}\right)-I\left(s_{k}\right)\right|. \end{array}$$

The principle of optimal segmentation is to make the divided target area and background area maintain the maximum similarity within the respective areas, while the similarity between the areas is kept to the minimum.

### 2.3. Microcalcification Research

#### 2.3.1. Definition

Microcalcifications (MCs) are a very important information for the imaging diagnosis of breast cancer. MCs are calcifications with a diameter of less than 1 mm on ultrasound or X-ray mammography, usually without acoustic shadow behind them. Microcalcification of breast cancer means that, during the treatment process, the patient has a certain degree of damage to the surrounding environment and human tissues, which in turn affects its function and causes local or systemic lesions. With the continuous proliferation, differentiation, and apoptosis of tumor cells, the volume of cancer foci gradually shrinks. There are a large number of tumor-causing factors (such as lymphoid binding protein) and microcalcification which reduce the activity of cellulolytic enzymes in the breast. At the same time, the pathological changes of breast cancer can also cause the cancer to enlarge and the surrounding tissues to be unevenly distributed throughout the human body, causing local or systemic lesions.

RETRACTED

#### 2.3.2. Research on the Correlation between Microcalcification and Mammary Glands

1. In terms of pathology, some scholars' studies have shown that the incidence of MCs in breast cancer histopathological examinations is 39% to 63%, and another researcher found that the incidence of MCs in breast cancer pathology research reports is even higher, up to 80%. The earliest pathologists believed that the formation of MCs in breast cancer tissue was mainly due to the rapid tumor growth leading to local cell avascular necrosis, resulting in dystrophic calcification. However, recent studies have shown that some cancer cells undergo stromal-like changes through specific procedures to obtain osteogenic function and then actively secrete osteogenic related proteins, hydroxyapatite, and calcium salts and jointly participate in the formation of MCs; the process is similar to bone formation.
2. The composition and imaging features of MCs are based on the oncology characteristics of breast cancer. Exploring the imaging features of MCs will have a great impact on the judgment of benign and malignant tumors and the assessment of breast cancer prognosis. The traditional view is that mammography is the gold standard for the diagnosis of breast cancer MCs. Breast ultrasound is susceptible to background noise, and MCs are often not well displayed. In the past, the imaging studies and clinical diagnosis of MCs used X-ray mammary glands.
3. However, as the understanding of breast cancer MCs continues to deepen, we urgently need an examination method that can accurately identify the nature of breast MCs at an early stage. Ultrasound technology should be the preferred inspection method due to its convenient, noninvasive, safe, and economical features. Compared with the hollow needle puncture technique guided by the molybdenum target, this method can significantly reduce the economic burden and physiological damage. Especially for in situ ductal carcinoma of the breast, the early imaging manifestations are only MCs. If surgical resection is performed as soon as possible, these patients are considered to be completely curable clinically, with the continuous improvement of high-frequency linear array probe technology, as well as the promotion of various new ultrasound-assisted diagnostic technologies, such as MicroPure imaging technology, speckle suppression technology, and breast three-dimensional ultrasound real-time imaging technology.

RETRACTED

Some researchers have reported that the sensitivity and specificity of ultrasound in the diagnosis of MCs can reach 95% and 88%, respectively. Some studies have confirmed that the sensitivity and specificity of MicroPure imaging technology to MCs are 70% and 30%, respectively.

#### 2.3.3. Chemical Composition of Breast Cancer MCs

Two types of MCs are commonly found in breast tissue. Type I is calcium oxalate (CaC2O4·2H2O) (HE staining) which does not stain, appears amber under the light microscope, and has a strong refractive index. It is difficult to observe by routine histological examination. It can only be observed with a polarizing microscope. It is captured. Type II is calcium phosphate, mainly in the form of HA. It appears off-white under light microscope, and the (HE) staining is alkaline blue staining. Some studies believe that the composition of the biochemical components of MCs is related to the disease state.

There are two types of breast calcification: large calcification and microcalcification. Large calcification is usually a degenerative change in the breast. The causes are mostly due to injury and inflammation, which is generally unrelated to cancer. Microcalcification may find calcium spots at the site of rapid decomposition of cells. These residues left by rapidly decomposing cells can be shown as microcalcification. When it appears in large numbers, it indicates the possibility of small tumors.

#### 2.3.4. Mechanism of Breast Cancer MCs

Current studies have found that there are two mechanisms for the formation of breast cancer MCs. Excessive proliferation of tumor tissue leads to ischemic necrosis of some cancer cells. The accumulation of a large number of acidic metabolites makes the cell microenvironment imbalance, proteases are denatured, necrotic cells cannot be degraded, and eventually necrotizing calcification is formed. The formation of breast cancer MCs may be a process mediated by cells. A part of breast cells undergo a specific process to transform from epidermal cell characteristics to mesenchymal cell characteristics under specific stimulation, thereby obtaining osteogenic function, secreting hydroxyapatite (HA), bone formation-related proteins (Bone Morphogenetic Proteins, (BMPs)), and other factors required for bone formation, as well as a large amount of transcription and expression of calcium channel protein to promote calcium ions into the cell, BMPs and their receptors enter the nucleus, localize to target genes, and then regulate under the synergistic effect of a series of signaling pathways, osteopontin (OPN), osteocalcin (OC), and other bone matrix proteins are expressed, and bone matrix proteins are deposited together with HA and calcium in cancer tissues, which ultimately leads to the formation of MCs.

RETRACTED

Therefore, this study used breast high-frequency ultrasound to analyze and classify the location, morphology, and distribution characteristics of breast cancer MCs and count the correlations with the diameter, pathological type, molecular type, and lymph node metastasis of breast cancer, in order to find a noninvasive imaging examination method to indirectly estimate the prognosis of breast cancer patients and to choose the right time and method for individualized treatment of breast cancer patients.

### 2.4. Prognostic Factors

The prognostic indicators of tumors include several aspects:

1. Clinical and pathological indicators: lymphatic metastasis, tumor size, tumor cell type, nuclear grade, etc.
2. Hormone receptor indicators, such as ER and PR
3. Molecular indicators
4. Other indicators, such as resistance to chemotherapy drugs

In addition, malignant epithelial tumor, also known as cancer, is the most serious disease endangering human health. In the United States, the mortality of malignant tumors is second only to cardiovascular disease. The first is malignant tumor, followed by cerebrovascular disease and heart disease. The most common and dangerous tumors are lung cancer, nasopharyngeal carcinoma, esophageal cancer, gastric cancer, colorectal cancer, liver cancer, breast cancer, cervical cancer, leukemia, and lymphoma.

In recent years, with the deepening of molecular biology and gene protein research, various molecular biological indicators related to the incidence and prognosis of breast cancer have been confirmed. Among the most commonly used molecular biological indicators are estrogen receptor ER, progesterone receptor PR, proto-oncogene human epidermal growth factor receptor-2, HER-2, and cell proliferation antigen marker Ki-67.

## 3. Experimental Investigation

### 3.1. Survey Object

Randomly perform contrast-enhanced ultrasound examinations on 100 female patients with breast cancer who were hospitalized in the People's Hospital from January to June 2021, and none of them received any treatment. The age of the patients is generally 23–69 years, with an average of 46.12 ± 11.50 years. The maximum diameter of breast cancer measured by ultrasound is 10–102 mm, with an average of 27.39 ± 18.14 mm.

RETRACTED

Note high safety and low side effects; microbubbles are uniform in size, less than 10 microns in diameter, and can be controlled. They can freely pass through capillaries and have hemodynamic characteristics similar to red blood cells; they can produce rich harmonics, with good stability. Ultrasound contrast agent must have the following conditions: being nontoxic and ultimately degradable or excreted from the body. It has strong scattering characteristics. Its diameter should be small enough to be smaller than the diameter of red blood cells (7 *μ*m), ensuring that it can enter the arterial circulation through the pulmonary capillaries, so as to achieve the imaging effect without causing embolism. It has sufficient stability and the retention time in the blood allows ultrasonic imaging to show the perfusion (enhancement) and clearance (regression) process in the tissue. It has clear damage threshold, predictability, and repeatability, can be removed quickly, and is easy to produce and easy to store, with suitable price.

### 3.2. Instruments and Inspection Methods

1. Ultrasound inspection uses Philips HD11 color Doppler ultrasound diagnostic apparatus, the probe is L12-3, and the frequency is 3–12 MHz. The molybdenum target inspection machine adopts GEMAXIRAY100TH-M1 molybdenum target machine.
2. Ultrasound examination of patients is done with the patients lying on their backs with hands raised to fully expose the bilateral breast and axilla. A series of transverse and longitudinal scans can be performed from top to bottom and from the inside to the outside. The examination speed is constant and sliding at a constant speed. Check the breasts on both sides, record the presence or absence of MCs, evaluate the location, shape, and distribution of the MCs lesions, and save the image data.

### 3.3. MCs Evaluation Criteria

1. Location: divided into inside the mass, outside the mass, and both inside and outside the mass
2. Morphology: divided into gravel-like calcifications with uniform particle size, usually less than 5 mm in diameter, densely distributed, and consistent gray scale, and non-gravel-like calcifications without such characteristics
3. Distribution: divided into clustered distribution, scattered diffuse distribution, and isolated distribution

### 3.4. Standards for Inspection Objects

#### 3.4.1. Entry Criteria

1. Female patients had primary invasive micropapillary carcinoma of the breast
2. The patients had not received systemic or local radiotherapy, chemotherapy, etc., before the diagnosis of the disease
3. Histopathological biopsy confirmed breast invasive micropapillary carcinoma (including pure type and mixed type)
4. The patient received standard breast cancer surgery: modified radical mastectomy or breast-conserving radical mastectomy and received the corresponding chemotherapy, radiotherapy, or endocrine therapy according to the corresponding clinical stage and molecular type after the operation
5. Patients gave informed consent

RETRACTED

#### 3.4.2. Exclusion Criteria

1. Male breast cancer patients
2. The case having a history of systemic or local radiotherapy or chemotherapy before the diagnosis
3. Histopathological biopsy diagnosis not containing invasive micropapillary carcinoma of the breast
4. Patients who have not undergone standardized breast cancer surgery in our center or who have not received corresponding individualized treatment after surgery
5. Incomplete clinical data or being lost to follow-up

### 3.5. Analysis Method

SPSS 20.0 statistical software was used for statistical description and analysis: qualitative data are expressed by frequency and percentage, differences between groups are compared by chi-square test, and comparisons between groups of data of various standard grades will be performed by rank-sum test.

Spearman rank correlation coefficient is used to describe the correlation between variables.

Logistic regression analysis is used to explore the influence of multiple factors of imaging parameters on prognostic indicators.

## 4. Result Analysis

### 4.1. Ultrasound Manifestations of Breast Cancer MCs and Pathological Classification of Breast Cancer

Among 100 patients with primary breast cancer, 84 were with invasive ductal carcinoma, 5 (4.8%) with in situ ductal carcinoma, 7 with mucinous carcinoma of the breast, and 3 with invasive micropapillary carcinoma of the breast. In the ultrasound findings of breast cancer, there was no significant statistical difference in the correlation between the location, shape, and distribution of MCs and the pathological classification of breast cancer; *p* position = 0.162, *p* shape = 0.18939, and *p* distribution = 0.197. The details are shown in Table 1.

### 4.2. Ultrasound Findings of Breast Cancer MCs Compared with the Diameter of the Cancer Focus

Among the 100 patients with primary breast cancer, 22 patients had cancer lesions less than 2 cm in diameter, 60 patients had cancer lesions between 2 cm and 5 cm in diameter, and 18 patients had cancer lesions greater than 5 cm in diameter. In the ultrasound findings of breast cancer, there was no significant statistical difference in the correlation between the location and distribution of MCs and the diameter distribution of cancer lesions; *p* position = 0.392 and *p* distribution = 0.798, there was a significant statistical difference in the correlation between MCs morphology and cancer lesion diameter; *p* form = 0.000; the specific situation is shown in Table 2.

RETRACTED

As shown in Figures 1–3, these figures, respectively, represent the comparison of the location, form, and distribution of the breast cancer MCs ultrasound appearance and the diameter of the cancer focus. In general, the diameter of the cancer foci is mainly at a distance of 2 to 5 cm. Among them, there were 5 cases in the grit-like calcification group with cancer foci greater than 5 cm in diameter and 13 cases in the non-gravel-like calcification group with cancer foci greater than 5 cm in diameter. There were 31 cases of tumors with a diameter of 2 to 5 cm in the mass and 31 cases of diffuse distribution.

### 4.3. Prognostic Indicators of Breast Cancer

In this paper, the prognostic indicators of breast cancer were tested experimentally, including tumor size, axillary lymph node metastasis, ER, PR, HER-2, and Ki-67, as shown in Table 3.

As shown in Figure 4, this is a picture of some prognostic indicators. We can know that there are 55 cases with tumors larger than 20 mm, 34 cases with axillary lymph node metastasis, 68% with ER positive, and 47% with PR negative.

## 5. Conclusion

The development of medical imaging technology not only provides a way to detect early clinically untouchable malignant tumors but also builds a platform to study the early natural development of breast cancer. Microcalcification is sometimes the only sign of breast cancer. The diagnostic value of ultrasound for breast cancer MCs has been controversial. In theory, high-frequency breast ultrasound has high resolution and the ability to detect MCs. However, in actual work, conventional ultrasound is not as good as X-ray in displaying MCs. Since the MCs signals are frequently masked by background noise, mammography cannot be highlighted. This largely limits the ultrasound diagnosis of breast cancer MCs. The presence of MCs indicates a poor prognosis of breast cancer. This conclusion has been confirmed by most studies. Compared with patients with primary breast cancer without MCs, patients with MCs have a larger tumor diameter and a higher rate of lymph node metastasis. Compared with the hollow needle puncture technique guided by the molybdenum target, the puncture method can significantly reduce the patient's economic burden and physical injury. With the development of computer technology and the wide application of computer vision principle, using computer image processing technology to detect and segment targets has become more and more popular. It should be widely used in medical treatment to reduce the burden of staff.

RETRACTED

## Figures and Tables

**Figure 1:** Comparison of MCs ultrasound performance of breast cancer and the location of cancer focal diameter.

**Figure 2:** Comparison of MCs ultrasound performance of breast cancer and the cancer focal diameter form.

**Figure 3:** Comparison of MCs ultrasound performance of breast cancer and the diameter distribution of cancer ranges.

**Figure 4:** Map of breast cancer prognosis indicators.

**Table 1:** Ultrasonic ultrasonography and pathological classification of breast cancer.

MCs ultrasound performance	IDC	DCIS	Mucinous carcinoma of breast	Breast invasive micropapillary carcinoma
Position				
Within the mass	51	1	2	1
Outside of the mass	10	3	3	0
The lump is inside and outside	23	2	2	2
Form				
Sand-like calcification	53	2	4	1
Non-sand-like calcification	31	4	4	2
Distribution				
Cluster distribution	24	2	4	1
Diffusion distribution	46	2	1	1
Isolated distribution	14	2	3	1

**Table 2:** MCs ultrasound of breast cancer was compared with focal diameter.

MCs ultrasound performance	<2 cm	2∼5 cm	>5 cm
Position			
Within the mass	12	31	8
Outside of the mass	2	9	4
The lump is inside and outside	8	20	6
Form			
Sand-like calcification	19	36	5
Non-sand-like calcification	3	24	13
Distribution			
Cluster distribution	8	21	5
Diffusion distribution	11	31	8
Isolated distribution	3	8	5

**Table 3:** Index status of breast cancer prognosis.

Prognostic indicator	Number of examples	Prognostic indicator	Number of examples
Mass size		PR	
≤20 mm	46	Yang	47
>20 mm	55	Yin	53
ARM lymph node metastasis		HER-2	
Yes	34	Yang	64
No	66	Yin	36)
ER		Ki-67	
Yang	68	Yang	71
Yin	32	Yin	29

## Data Availability

The data underlying the results presented in the study are included within the manuscript.

## References

[1] Zhou C., Liu J., Gou B., Hu J., Huang R. (2020). Ultrasound BI-RADS sign analysis of different molecular types of breast cancer and its correlation study. *Cancer Prevention and Treatment*.

[2] Zhu Y., Nie F., Lu W. (2020). Correlation study between the features of conventional ultrasound and contrast-enhanced ultrasound and the expression of HER-2 in breast cancer. *Chinese Journal of Ultrasound in Medicine*.

[3] Li D., Chen W. (2020). Study on the correlation between breast cancer microcalcification and the expression of ER, PR and HER-2. *Journal of Liaoning Medical College*.

[4] Geng Y., Leng X., Song Y. (2020). Correlation between breast background ultrasound classification and histological and morphological features of breast cancer. *Chinese Journal of Clinical Medical Imaging*.

RETRACTED

[5] Wu S. (2019). Study on the correlation between clinicopathology and ultrasound imaging characteristics of invasive breast cancer. *Electronic Journal of Modern Medicine and Health Research*.

[6] Ye Y. (2020). Study on the correlation between ER, PR, CerbB-2 and breast cancer ultrasound images. *Chinese Health Standard Management*.

[7] Guo T. (2019). Correlation analysis of breast cancer microcalcification and prognosis. *China Rural Health*.

[8] Cai W., Sun Y. (2019). Comparison and combined application analysis of ultrasound and mammography in breast cancer examination. *Journal of Shenyang Medical College*.

[9] Tang T. (2019). A related study on the pathological types of breast cancer with microcalcifications in the ultrasound image. *China Practical Medicine*.

[10] Zhou C., Wang X., Li X. (2019). Study on the correlation between the characteristics of enhanced ultrasound imaging and prognostic factors in breast cancer. *Chinese Journal of Clinical Medicine*.

[11] Duan J., Zhao C., Wang X. (2019). Analysis of ultrasound signs and prognostic factors of breast cancer microcalcification. *Chinese Medicine*.

[12] Wu S., Ouyang Y., Cui B. (2020). Review of ultrasound detection methods for breast microcalcification. *Journal of Beijing University of Technology*.

